# Correlation between 25-Hydroxyvitamin D, sFlt-1, PLGF, and Hypertension in Pregnancy

**DOI:** 10.1155/2021/9371953

**Published:** 2021-11-01

**Authors:** Wei Wang, Ting Du, Xiaoqi Jiang

**Affiliations:** Obstetrics Department, Weifang Maternal and Child Health Hospital, Weifang 261000, Shandong, China

## Abstract

Gestational hypertension is a common disease in clinical practice, which does great harm to the mother and infant. The purpose of this study was to investigate the relationship between 25-hydroxyvitamin D, sFlt-1, and PLGF and hypertensive disorder complicating pregnancy. Specimen preparation: after delivery or placental caesarean section, in order to avoid calcification and necrosis in the middle of the placenta, an area of about 1.5 cm × 1.5 cm × 1.5 cm should be separated immediately. After dehydration, use a Citadel 2000 dryer to dry it and place it in a block of saline for xylene immunohistochemical staining. Statistical processing was performed according to the proportion of positive cells in each part and the depth of staining. Placental tissue collection and treatment: within 20 minutes after the delivery of the placenta, two pieces of the placental tissue (about 1.0 cm × 1.0 cm × 1.0 cm) were taken from the central zone of the placental maternal surface without obvious bleeding and calcification. They were rinsed repeatedly in normal saline, fixed in 10% neutral formaldehyde solution for 24 hours, dehydrated using an automatic dehydrator, and embedded in paraffin for detection. Before the study, 20 ml of distilled water was added to the sample to stand for 20 minutes; the Cobas E610 immunoanalyzer was turned on, and sFlt-1 and PLGF (placental growth factor) were selected. The serum 25-hydroxyvitamin D level of pregnant women was detected in the fasting state at 24–28 weeks of gestation, and the best collection time was 8 : 00–11 : 00 in the morning. 5 ml of the whole blood sample without anticoagulant was collected and stored at 0–4°C in a cold storage and dark environment. The serum was obtained by high-speed centrifugation within 24 hours after collection. The method is suitable for the quantitative determination of 25-OH-vitamin D in human serum. In the hypertensive pregnancy group, the level of 25-hydroxyvitamin D was 18.44 ± 3.48 ng/ml, and the sFlt-1/PLGF level was highest at 0–5 weeks followed by 5–10 weeks, 10–15 weeks, and 15–20 weeks. This study provides new ideas and experimental clues for the prevention and treatment of pre-eclampsia.

## 1. Introduction

So far, the etiology and mechanism of hypertension in pregnancy have not been fully elucidated. At present, it is believed that its pathogenesis is mainly related to superficial placental implantation, genetic factors, maternal-fetal immune balance imbalance, vascular endothelial damage, blood coagulation and fibrinolytic system imbalance, and genetic susceptibility. Sensitivity, oxidative stress, nutritional disorders, and insulin resistance are related. Therefore, it is necessary to find effective predictive indicators and prevent the occurrence of hypertensive disorder as soon as possible; it has become a new research field and hotspot in recent years. Hypertension in pregnancy is a common complication in obstetrics. Foreign statistics show that the disease accounts for 5% to 10% of all pregnancies, and the domestic incidence rate is 5% to 12%, including hypertension during pregnancy, pre-eclampsia, eclampsia, pregnancy combined with chronic hypertension, and chronic hypertension complicated with pre-eclampsia, the first three are pregnancy-induced hypertension (PIH), which refers to the occurrence after 20 weeks of pregnancy, with hypertension, proteinuria, and/or edema are the main clinical symptoms, convulsions and coma may occur in severe cases, and all symptoms disappear within 12 weeks after delivery.

In this way, new serological prediction standards can be found to be able to early and objectively evaluate the progress of the disease and evaluate the prognosis, detect abnormalities in time, and take preventive measures early to better and more effectively guide clinical diagnosis, treatment, and prevention, so as to maximize the guarantee. Mother and child safety reduce the occurrence of complications such as intrauterine growth retardation, cardiovascular and cerebrovascular accidents, liver and kidney damage, placental abruption, premature delivery, intrauterine fetal death, and amniotic fluid embolism in order to achieve a relatively ideal pregnancy outcome, which not only for the majority of patients with hypertension in pregnancy bring well-being but also have important guiding significance for the diagnosis, treatment, and prevention of the disease in obstetrics. Due to vasospasm, increased blood pressure, increased peripheral resistance, increased myocardial contractility and ejection resistance, and ventricular function in a hyperdynamic state, patients with hypertension in pregnancy suffered cardiac insufficiency. Therefore, monitoring the BNP of such patients in clinical practice is necessary. In practice, the observation of the condition of hypertension in pregnancy has certain guiding significance, and it has certain significance in assessing myocardial damage in patients with hypertension in pregnancy.

In patients with idiopathic pulmonary hypertension (IPAH), disease progression and survival are related to the ability of the right ventricle to adapt to chronic pulmonary hypertension. Ghio believes that although some echocardiographic variables have been correlated with prognosis in previous studies, all right ventricular (RV) function indexes available on echocardiography have never been compared and evaluated. In his research, the degree of tricuspid regurgitation, the foldability of the inferior vena cava, the flow pattern of the superior vena cava, and the left ventricular diastolic eccentricity can be determined, but the relationship between the left ventricular eccentricity index and the prevalence is not mentioned [1]. The purpose of Vidal's study is to determine the epidemiology and prognosis of intra-abdominal hypertension in heterogeneous intensive care unit populations. His research was conducted in the surgical intensive care unit of the university hospital. His study patients included all patients who had been admitted to the hospital continuously within 9 months, had a hospital stay of >24 hours, and required bladder catheterization. At the time of admission, the epidemiological data and risk factors of intra-abdominal hypertension were studied; then, daily maximum and average intra-abdominal pressure (IAP (maximum) and IAP (average)) and intraperitoneal perfusion pressure were recorded. Fluid balance, filtration gradient, and continuous organ failure assessment score were also recorded. His research involved the definition of intra-abdominal hypertension and the signs of new organ failure but did not make a multisample analysis [2]. Dodick believes that the clinical syndromes of hypertension, headache, palpitation, sweating, flushing, and emotional instability are usually related to pheochromocytoma. Two patients in his study showed these symptoms, but pheochromocytoma was not found. Although after the combined use of several antihypertensive drugs the unstable fluctuations of blood pressure and headache could not be controlled, a rapid and long-lasting response appeared after the administration of clonidine. Although he reviewed the pathophysiology of the syndrome and the mechanism of action of clonidine under the background that the baroreflex may fail, the research process lacked comparative data [3]. Abdulsalam believes that idiopathic intracranial hypertension (IIH) is a neurological disease characterized by increased intracranial pressure without potential intracranial pathological changes. He believes that this disease is rare in men and is mainly seen in obese women of childbearing age. An interesting case of IIH occurred in a male patient. The male patient developed severe vision loss within 2 weeks and was successfully treated with surgery. Therefore, in men with rapidly progressive vision loss, surgical intervention should be considered as early as possible. Further prospective studies are needed to evaluate the role of early surgical intervention and drug therapy in this group of patients. Although IIH is less common in men than in women, men are more prone to vision loss, which is usually severe and less responsive to medication [4].

This study mainly explored the correlation between 25-hydroxyvitamin D, sFlt-1, and PLGF and hypertension in pregnancy. This study provides new ideas and experimental clues for the prevention and treatment of pre-eclampsia.

## 2. Hypertension during Pregnancy

### 2.1. Hypertension Disease

With the continuous development of the high-efficiency rhythm of society, people's health concerns and awareness of prenatal and postnatal care are generally improved. How to predict the condition of hypertension in pregnancy, one of the four major causes of maternal death, and make effective treatments in time? To ensure the safety of mothers and children to the greatest extent and reduce the occurrence of critical complications to achieve a relatively ideal pregnancy outcome has become an urgent problem [5, 6]. Although the study of the etiology and mechanism of this disease has always been an important subject in obstetrics, scholars at home and abroad have also done a lot of research on its etiology and pathogenesis. The previous descriptions of the etiology of hypertension in pregnancy mainly include immune mechanism, genetic factors, abnormal expression of endothelial nitric oxide synthase, superficial infiltration of uterine placental trophoblast cells, uterine spiral artery recasting disorder leading to uterine placental ischemia, abnormal performance of some cytokines, gene mutations or genetic polymorphisms, inflammation, blood vessels and endothelial cells damage, and other reasons, but the specific pathogenesis has not yet been clearly definitive [7]. In recent years, the theory of vascular endothelial injury has become a hot research topic at home and abroad, and it is recognized as one of the main causes of hypertension in pregnancy [8, 9].

The short-term energy calculation of the signal at time *n* is defined as follows [10]:

(1) $$\begin{array}{c} E_{n}={\sum_{m=-\infty }^{\infty }\left[x\left(m\right)\cdot w\left(n-m\right)\right]}^{2}. \end{array}$$

Among them, *E*_*n*_ is the energy value [11].

(2) $$\begin{array}{c} R\geq \left(1-\frac{q_{ppk}}{q_{H_{1}}}\right)\left(1-\frac{q_{att}}{2^{l}}\right)\left(1-\frac{q_{sc}\left(q_{H_{2}}+q_{H_{3}}\right)}{2^{l}}\right)\varepsilon . \end{array}$$

Here, *R* is the total amount of data transmission for data transmission [12].

(3) $$\begin{array}{c} P_{i,j}=\exp\left(\frac{\alpha_{i}D_{HOL}-x}{1+\sqrt{x}}\right),\\ K_{c}=\frac{1}{L}\sqrt{\sum_{i=0}^{l-1}{\left[y\left(k-i\right)-y_{m}\left(k-i\right)\right]}^{2}+y_{m}\left(k-i\right)}. \end{array}$$

Here, *P*_*ij*_ represents the final delayed power. The average gray scale of regions *A* and *B* is determined using the below equation [13]:

(4) $$\begin{array}{c} \mu_{A}=\frac{1}{\omega }\sum_{i=1}^{k}i*p_{i}\\ =\frac{\mu \left(k\right)}{\omega \left(k\right)},\\ \mu_{B}=\frac{1}{\omega }\sum_{i=k+1}^{L}i*p_{i}\\ =\frac{\mu -\mu \left(k\right)}{1-\omega \left(k\right)}. \end{array}$$

Among them, *μ* is the average gray level of the whole image [14].

(5) $$\begin{array}{c} \mu =\sum_{i=1}^{L}i*p_{i}\\ =\omega_{A}\mu_{A}+\omega_{B}\mu_{B}. \end{array}$$

The variance of the two regions is calculated using the below equation [15, 16]:

(6) $$\begin{array}{c} \sigma^{2}=\omega_{A}{\left(\mu_{A}-\mu \right)}^{2}+\omega_{B}{\left(\mu_{B}-\mu \right)}^{2}\\ =\frac{\mu \omega \left(k\right)-\mu \left(k\right)}{\omega \left(k\right)\left(1-\omega \left(k\right)\right)}. \end{array}$$

### 2.2. 25-Hydroxyvitamin D

Serum 1,25(OH)2D3 content is stable, and serum or plasma 25-hydroxyvitamin D3 (25(OH)D3) is currently a relatively recognized indicator for evaluating vitamin D levels [17]. It can reflect the amount of vitamin D ingested from foods (including supplementary foods and vitamin D-fortified foods) through skin exposure to ultraviolet rays. Some people believe that low vitamin D levels in the first trimester lead to the occurrence of pre-eclampsia. Because the symptoms of pre-eclampsia occur earlier than the appearance of pre-eclampsia, the controversy is mainly due to the fact that most trials only collect data during the first or third trimester of pregnancy, and there is a lack of systematic pregnancy. Correlation analysis of vitamin D changes during the whole pregnancy from early to third trimester. In addition, most domestic and foreign studies have focused on the correlation between vitamin D and pre-eclampsia, but there are fewer studies analyzing hypertension during pregnancy. Although the harm of hypertension during pregnancy is less than the former, if its related risk factors can be found, early intervention and early diagnosis and treatment can effectively prevent disease development and improve prognosis [18, 19].The molecular structures of 25-hydroxy vitamin D3 and 25-hydroxy vitamin D2 are shown in Figure 1.

### 2.3. PLGF and sFlt-1

Hypertensive disorders suffered by women during pregnancy are collectively referred to as hypertensive disorders in pregnancy (HDCP) [20]. The molecular structure of PLGF is a glycoprotein homodimer molecule, and its protein amino acid sequence has 46% homology with VEGF [21]. The selective splicing of PLGF by mRNA can produce different protein subtypes: PLGF1, PLGF2, and PLGF3. PLGF2 is different from the other two subtypes. It contains a region of 21 basic amino acids and has heparin-binding activity like VEGF2. The receptors of PLGF and its mediated biological functions have two types of tyrosine kinase receptors of VEGF family: VEGFR1/Flt1 and KDR/Flt1. The biological function of PLGF is activated by specifically binding its receptor VEGFR1/Flt1. VEGFR1/Flt1 has a strong biological activity. It can mediate the effect of endothelial cells and stromal cells when combined with its ligands and also affect the differentiation and maturation of endothelial cells. When Flt1 is defective, a lot of accumulation of endothelial cells can be formed, but new blood vessels cannot be formed [22, 23]. It shows that Flt1 is related to maintaining the adhesion between endothelial cells and endothelial cells, and between endothelial cells and matrix, and maintaining vascular permeability.

PLGF is related to the occurrence of hypertension in pregnancy (HDCP) and “placental superficial implantation”. The decreased expression of PLGF may also be a factor affecting shallow implantation of the placenta. Impaired trophoblast infiltration capacity and decreased maternal vascular turnover eventually lead to reduced placental blood vessel formation, placental bed ischemia, and hypoxia [24], destroying normal trophoblast cell function and endothelial cell proliferation, which are related to the occurrence of pregnancy-induced hypertension in pre-eclampsia. The absolute center frequency is used to calculate the value of the absolute center frequency of the EEG signal [25].

(7) $$\begin{array}{c} ACF=\left|CF_{\alpha }-CF_{b}\right|. \end{array}$$

Among them, *CF* represents the center frequency of the point*α*. The relative center frequency is used to calculate the value of the EEG signal relative to the center frequency [26, 27].

(8) $$\begin{array}{c} RCF=CF_{\alpha }-CF_{b}. \end{array}$$

The slope is used to calculate the value of the slope of the EEG signal [28].

(9) $$\begin{array}{c} \text{Slope}=\tan\;\alpha \\ =\frac{h}{d}\times 100\%. \end{array}$$

The brain waves of nearby pixels generally have a high degree of spatial correlation. That is, adjacent pixels with similar attributes are divided into classes with the same probability. The spatial information of image segmentation is very important, but it means that traditional algorithms do not need to consider the spatial correlation of blurred pixels [29, 30].

(10) $$\begin{array}{c} J_{m}=\sum_{i=1}^{c}\sum_{j=1}^{N}u_{ij}^{m}{\left\|x_{j}-v_{i}\right\|}^{2}+\frac{\alpha }{N_{R}}\sum_{i=1}^{c}\sum_{j=1}^{N}u_{ij}^{m}{\left\|x_{r}-v_{i}\right\|}^{2}. \end{array}$$

When performing data statistics on a single specimen:

(11) $$\begin{array}{c} N={\left[\frac{Z_{1}\sqrt{\pi \left(1-\pi \right)\left(Q_{1}^{-1}+Q_{2}^{-1}\right)}+Z_{2}\sqrt{\pi \left(1-\pi \right)\left(Q_{1}^{-1}+Q_{2}^{-1}\right)}}{\pi_{1}-{}_{\pi }^{2}}\right]}^{2}. \end{array}$$

Among them, *N* is the number of samples. Solve the estimated value.

(12) $$\begin{array}{c} \ln\left(\frac{P{}^{\prime }/1-P{}^{\prime }}{p/1-p}\right)=\beta_{1}\left(x_{1}-x_{2}\right)+\beta_{2}\left(x_{2}-x_{3}\right)+\cdots +\beta_{n}\left(x_{n-1}-x_{n}\right). \end{array}$$

Perform image correlation coefficient *β* analysis.

(13) $$\begin{array}{c} \log\;p=\ln\frac{p}{1-p}=\beta_{0}+\beta_{1}x_{1}+\beta_{2}\left(x_{2}^{\prime }-x_{2}\right)+\cdots +\beta_{n}\left(x_{n}^{\prime }-x_{n}\right). \end{array}$$

The introduction of real-time three-dimensional echocardiography (RT-3DE) has revolutionized echocardiography technology [31]. Hypertension in pregnancy is a unique disease during pregnancy. Its occurrence may be related to shallow placental implantation, dysplasia of the placental vascular network, and placental ischemia and hypoxia. PLGF is mainly secreted by trophoblast cells and vascular endothelial cells. PLGF has important paracrine and autocrine effects on angiogenesis and trophoblast cell infiltration. Therefore, it is speculated that PLGF and F1t1 may be abnormally expressed in HDCP, and PLGF and Flt1 are affected by it. Body binding may affect the production of NO, and PLGF may play a role in the pathogenesis of HDCP by affecting the level of NO [32].

## 3. Experiments on Related Factors of Hypertension during Pregnancy

### 3.1. Research Objects and Standards

Serum was collected from pregnant women in the obstetric outpatient, emergency, ward, or hospitalization of our hospital from January 2019 to May 2019, including pregnant women with pre-eclampsia who had clinical onset after 20 weeks and pregnant women with normal blood pressure who gave birth from 10 weeks to term. The study was appraised by the ethics committee, and all research subjects signed the “Informed Consent” form.

Cases with complete clinical data were included. It is a prospective case-control study including pregnant women who underwent a caesarean section before giving birth to the first child; the diagnostic criteria of hypertension during pregnancy were based on the Classification of the Sixth Edition of “Obstetrics and Gynecology”. There was no premature rupture of membranes and premature rupture of membranes in each group. *Signs of infection*. All cases had no other obstetric complications and primary liver and kidney complications. There were no statistically significant differences in the number of pregnancy, gestational age, and basal systolic blood pressure and diastolic blood pressure of each component (*P* > 0.05).

*Case selection criteria*. (1) age 18–40; (2) no serious medical and surgical complications before pregnancy; (3) no family history of hypertension, diabetes, heart disease, and other diseases; (4) this pregnancy was a singleton pregnancy; (5) liver and kidney function and thyroid function are normal.

*Case exclusion criteria*. (1) age <18 or >40 years; (2) severe medical and surgical complications before pregnancy; (3) family history of hypertension, diabetes, heart disease, and other diseases; (4) the pregnancy was multiple births pregnancy; (5) abnormal liver and kidney function and thyroid function.

### 3.2. Main Reagents

  sFlt-1 working solution (kit). Product number: 05109523190, batch number: 15418501 and 15568401.
  PLGF working solution (kit). Product number: 05144671190, batch number: 15418601 and 15470001.

### 3.3. Specimen Preparation

After delivery or placental caesarean section, in order to avoid calcification and necrosis in the middle of the placenta, an area of about 1.5 cm × 1.5 cm × 1.5 cm should be separated immediately. All samples washed with normal saline will remain 10% static. After dehydration, use a Citadel 2000 dryer to dissolve the formaldehyde solution and embed it in a block of saline for xylene immunohistochemical staining. Soak the sulfuric acid solution in sulfuric acid emulsion for more than 24 hours, rinse the sulfuric acid solution with running water, soak in 95% ethanol for 24 hours, and rinse with distilled water 3–5 times. Place the slides and dry them in the oven. Adhesive treatment: dilute APES with pure acetone 1 : 150, soak the slide for 1 to 2 minutes, take it out, and dry at 37°C at low temperature. The paraffin-covered block was sliced continuously with an AS-325 slide, and the thickness of the slice was 5 *μ*m. Dehydrate regularly. Then, add 3% hydrogen peroxide (H_2_O_2_) and heat at room temperature for 10–15 minutes. Rinse with distilled water 3 times and draw wax edges. Add 0.1 mmol/L of phosphate-buffered saline (PBS) (pH 7.2–7.4), boil at 98–100°C for 20 minutes, and then cool to room temperature.

### 3.4. Results Judgment

Statistical analysis was carried out according to the proportion of positive cells in each part and the depth of staining. Positive cell staining judgment: <5% is 0, 5%–25% is 1, 26%–50% is 2, and >50% is 3. Positive intensity: when the original state score is 0, there are no yellow positive particles in the cell; when the state score is 1, some light yellow particles can be seen in the nucleus or cytoplasm; when the state score is 2, a lot of dark brown particles can be seen; when the status score is 3, these cell particles can be clearly seen. Scores are based on the points of the two indicators. Points 0 is −, 1–3 is +, 4–6 is ++, and 7–9 is +++.

### 3.5. Collection and Determination of sFlt-1 and PLGF and 25-OH-VitaminD

#### 3.5.1. Collection and Processing of sFlt-1 and PLGF Specimens

(1) Serum collection and treatment: the subjects in each group were drawn 6.0 ml of cubital venous blood on an empty stomach early in the morning before delivery; put it in a common test tube and let it stand for 1 hour, dissociate the heart for 20 minutes at 3000 rpm/min, collect the serum, and place it in a sterile Eppendorf tube, frozen at −70°C for testing.
(2) Placental tissue collection and processing: within 20 minutes after the placenta was delivered, at the central zone of the maternal surface of the placenta without obvious hemorrhage and calcification, take 2 pieces of placental tissue about 1.0 cm × 1.0 cm × 1.0 cm and rinse them repeatedly in saline, clean, fix in 10% neutral formaldehyde solution for 24 hours, and embed in paraffin after being dehydrated using an automatic dehydrator for testing.
(3) 24-hour urine output collection and processing of patients with pre-eclampsia (mild and severe): before delivery, collect urine for 24 hours (from 8 am to 8 am the next day), and accurately record the urine output at 9 am the next morning. Take 10 ml of it and send it to the laboratory for processing.
(4) Detection steps:
  ① Add 20 ml of distilled water to the sample before the study and let it stand for 20 minutes for inspection
  ② Turn on the Cobas E610 immunoassay analyzer
  ③ Place the solution reagent glass tube on the solution reagent glass tube rack in order, and then the Cobas E610 immunoassay analyzer will automatically read the reagent related information by scanning the barcode on the side of the solution reagent glass tube.
  ④ Select the test items sFlt-1 and PLGF
  ⑤ Quality control: arrange the samples to be tested in the order of the sample racks; select QC from the test request menu; select the quality management items as sFlt-1 and PLGF, and then enter the number of the sample rack and the position on the sample rack. Configure various levels of quality management projects. Because quality management items do not have barcodes, you need to manually enter the target values and ranges of the quality management items.
  ⑥ Calibration: put the calibration fluids in order on the calibration rack; select “Calibration” under the test request menu; select the calibration items as sFlt-1 and PLGF, and then enter the number of the calibration rack placed on the calibration fluid of different levels and position on the calibration frame. The instrument automatically completes the detection and corrects the preset calibration curve according to the measured calibration concentration to complete the calibration.

The quality calibration of PLGF and sFlt-1 is shown in Table 1.

#### 3.5.2. Collection and Determination of 25-OH-VitaminD

1. Collection
2. Collection method: when pregnant women who met the inclusion criteria are discharged from the hospital, one-on-one guide them to fill in the collection, and then the relevant data will be collected. The serum 25-hydroxyvitamin D level of pregnant women was tested in the morning when the pregnant women were 24–28 weeks of gestation. The best collection time was 8 : 00–11 : 00 in the morning. Collect 5 ml of the whole blood sample without anticoagulant, place it in a refrigerator and dark environment at 0–4°C after collection, and centrifuge at high speed within 24 hours after collection to obtain serum. The content of 25(OH)D in serum samples was detected by liquid chromatography-mass spectrometry LCMS/MS, and the test report was issued by the medical laboratory of our hospital.
3. Scope of application: this method uses liquid chromatography-mass spectrometry, which is suitable for the quantitative determination of 25-OH-VitaminD in human serum. This method can accurately reflect the level of 25-OH-VitaminD in the serum samples to assist in the diagnosis of related diseases.
4. Test principle: after the serum sample has been subjected to pretreatment processes such as protein removal and extraction, the unknown interfering substances that may interfere with it are separated through the chromatographic column and detected by LCMS/MS, the concentration of the solution corresponding to the ratio of the peak area of vitamin D to the peak area of the internal standard was used to make a standard curve to calculate the serum vitamin concentration, and the internal standard method was used to quantify vitamin D in the sample, which is quantified by the internal standard method.
5. Sample storage: 5 ml of whole blood sample without anticoagulant should be placed in a refrigerator and dark environment at 0–4°C after collection, and the serum should be centrifuged within 24 hours after blood collection.
6. Specimen collection: the vitamin D serum concentration (VitD) was monitored. Serum specimens were collected in red cap/yellow cap separation gel specimen collection tubes.
7. Specimen rejection criteria: specimen identification is unknown; serum specimens are less than 1 ml; hemolysis, chyle, etc., occur.
8. Presampling requirements: Vitamin D (VitD); fasting with vitamin D-rich health products and medicines for at least 1 day before collecting the specimens.
9. Diagnostic criteria for serum 25-hydroxyvitamin D (25(OH)D) levels
10. At present, there is controversy about the reference value range of vitamin D. According to the kit instructions and the standards adopted in most documents, the reference ranges of this study are as follows: lack, serum 25(OH)D level < 20 ng/ml; insufficient, 20 ≤ serum 25(OH)D level < 30 ng/ml; normal, 30 ng/ml ≤ serum 25(OH)D level ≤ 100 ng/ml; overdose, serum 25(OH)D level > 100 ng/ml.

## 4. Results and Discussion

### 4.1. Research Sample Analysis

2008 people were included in the study and collected blood samples from the first trimester. In the end, 78 people had hypertension during pregnancy, 46 had pre-eclampsia, 37 had severe pre-eclampsia, 0 had eclampsia, and 1641 had normal pregnancy. In normal pregnant women, 200 people were randomly selected as controls. The basic information of the research object was expressed by the mean value ± standard deviation, and the differences between the groups were compared by analysis of variance. The results showed that there were no significant differences in age, pregnancy times, pre-pregnancy body mass index (BMI), and gestational age of blood collection among the groups (*P* > 0.05). The basic information of the research object is shown in Table 2.

### 4.2. Correlation Analysis of Hypertension during Pregnancy

At 12–18 weeks of gestation, the mean serum 25(OH)D level in the normal pregnant women group was 19.33 ± 4.75 ng/ml; the hypertension group during pregnancy was 18.44 ± 3.48 ng/ml, with mild eclampsia; the pre-eclampsia group was 12.29 ± 2.79 ng/ml; and the severe pre-eclampsia group was 9.56 ± 2.68 ng/ml. There was no significant difference in the mean serum level between the pregnancy-induced hypertension group and the normal pregnant group (*P* > 0.05) At 30–36 weeks of pregnancy, the mean serum 25(OH)D levels of each group were 22.57 ± 4.33 ng/ml, 20.09 ± 3.38 ng/ml, 18.68 ± 3.50 ng/ml, and 9.48 ± 2.98 ng/ml, respectively. The difference between the hypertensive disease group during pregnancy and the normal pregnancy group was statistically significant (both *P* < 0.05), and with the gradual aggravation of hypertension during pregnancy, the level of 25-hydroxyvitamin D showed a downward trend. The correlation analysis of hypertension during pregnancy is shown in Figure 2.

The serum 25(OH)D levels of each group are shown in Table 3. The serum 25(OH)D level of each group is expressed as mean ± standard deviation, and the serum 25(OH)D level in the first trimester of A, B, C, and D groups are, respectively, 17.47 ± 6.41 ng/ml, 14.33 ± 5.60 ng/ml, 11.26 ± 4.54 ng/ml, and 18.21 ± 6.73 ng/ml. Serum 25(OH)D levels in the third trimester of pregnancy were 20.66 ± 7.06 ng/ml, 16.54 ± 6.51 ng/ml, 13.03 ± 5.79 ng/ml, and 21.04 ± 7.63 ng in groups A, B, C, and D, respectively.

In this study, we used immunohistochemistry, western blotting, and RT-PCR to determine the placental PLCF, Flt-1 protein, and mRNA in the normal pregnancy group (control group) and HDCP groups. The expression of PLCF in the placenta of the severe group was significantly lower than that of the control group (*P* < 0.05). It is suggested that HDCP may change the morphology and function of trophoblast cells due to placental ischemia and hypoxia, which can cause downregulation of PLCF secretion, and low PLGF levels will affect the proliferation and infiltration capacity of extravillous trophoblast cells in HDCP patients and interfere with the fetal placenta. The normal blood vessel network is formed, which further develops the hypoxia of the placenta. Flt-1 protein immunohistochemical staining is shown in Figure 3.

The content of sFlt-1 in different periods is shown in Figure 4. It can be seen intuitively from Figure 4 that during the early and second trimester, the level of sFlt-1 (soluble fms-like tyrosine kinase-1) in serum does not change significantly. After the third trimester, the sFlt-1 level is elevated, especially after the full term. The levels of sFlt-1 at different stages were analyzed by variance analysis, and Dunnett's T3 test was used for multiple comparisons between groups. Compared with the four stages 0–5, 5–10 weeks, 10–15 weeks, and 15–20 weeks, there was no significant difference in the sFlt-1 level between the groups, all of which were *P* > 0.05. Among them, the level of sFlt-1 at 15–20 weeks was relatively low; the sFlt-1 levels increased after 20–25 weeks and 30 weeks, compared with 10–20 weeks, the difference was significant (*P* < 0.05); after 37 weeks, compared with the other groups, the sFlt-1 level increased significantly high (*P* < 0.001).

The single-factor analysis of variance showed that the difference between the serum PLGF levels of pregnant women in the normal pregnancy group, mild pre-eclampsia group, and severe pre-eclampsia group was statistically significant, indicating that the normal pregnancy group and the mild pre-eclampsia group were statistically significant. The serum PLGF levels of pregnant women are different between the prepurpura group and the severe prepurpura group. Pairwise comparison (SNK test) is required to confirm the differences between groups. The expression of PLGF in humans is shown in Figure 5.

Figure 6 shows the analysis of PLGF (placenta growth factor) levels at different stages. At 0–5 weeks, the PLGF level is the lowest followed by 5–10 weeks, 10–15 weeks, and 15–20 weeks, and then the PLGF level increased significantly (*P* < 0.001); there was no significant difference between the three groups 20–25 weeks, 25–30 weeks, and >30 weeks, all of which were *P* > 0.05. At 20–25 weeks, the level was highest. After 37 weeks, the PLGF level was significantly reduced (*P* < 0.05). The reasons for the decrease in PLGF content during hypertension in pregnancy may include insufficient infiltration of maternal spiral artery trophoblast cells in the first trimester, increased glomerular capillary permeability, PLGF leakage through capillaries resulting in increased loss, and hypoxia. The expression is downregulated, and the metabolic rate is increased.

Figure 7 shows the analysis of the ratio of sFlt-1/PLGF at different stages. The ratio was highest at 0–5 weeks and then gradually decreased at 5–10 weeks, 10–15 weeks, and 15–20 weeks. There were significant differences between the adjacent two groups, with *P* < 0.05. At 28–32 weeks and 33–36 weeks, the ratio increased slowly than before, but the difference was not significant. After 37 weeks, it increased significantly compared with 33–36 weeks (*P* < 0.05).

## 5. Conclusion

Hypertension during pregnancy is a common disease in clinical practice, which is extremely harmful to mothers and babies. This study mainly explored the correlation between 25-hydroxyvitamin D, sFlt-1, and PLGF and hypertension in pregnancy. This method uses liquid chromatography-mass spectrometry and is suitable for the quantitative determination of 25-OH-VitaminD in human serum. This study provides new ideas and experimental clues for the prevention and treatment of pre-eclampsia. In summary, the abnormal expression of PLGF, sFlt-1, and Flt-1 plays an important role in the pathogenesis of hypertension in pregnancy. The imbalance of sFlt-1/PLGF regulation axis may be involved in the pathogenesis of hypertension in pregnancy. sFlt-1 can be used as a marker for the detection of skin cell damage in pre-eclampsia during pregnancy-induced hypertension. It can also be used to observe its content to infer the severity of the disease, which is important for timely termination of pregnancy and reduction of maternal and infant complications. Clinically, if we can dynamically observe the changes of PLGF, sFlt-1, and Flt-1 content, it may play an important role in guiding the treatment of hypertension in pregnancy.

## Figures and Tables

**Figure 1:** 25-Hydroxy vitamin D3 and 25-hydroxy vitamin D2 molecular structure (http://alturl.com/xgvaz)(http://alturl.com/5f74f).

**Figure 2:** Correlation analysis of hypertension during pregnancy.

**Figure 3:** Flt-1 protein immunohistochemical staining (http://alturl.com/5d2cx).

**Figure 4:** The content of sFlt-1 in different periods.

**Figure 5:** Expression of PLGF in human body (http://alturl.com/rzwh8).

**Figure 6:** Analysis of PLGF (placenta growth factor) levels at different stages.

**Figure 7:** Analysis of the ratio of sFlt-1/PLGF at different stages.

**Table 1:** PLGF and sFlt-1 quality calibration.

Parameter	sFlt-1		PLGF	
	1	2	1	2
Target value	881	9100	77.8	1840
Range	620–1151	6615–12285	59.7–111	l 260–2340
Measured	883.4	9159	77.08	1876

**Table 2:** Basic information of research objects.

Group	N	Pregnancy times (times)	Gestational week of blood collection in the first trimester (weeks)	Gestational week of blood collection in the third trimester (week)	BMI before pregnancy (kg/m^2^)
Normal pregnancy	200	1.98 ± 0.97	10.94 ± 1.26	34.13 ± 1.02	21.55 ± 1.47
Hypertension during pregnancy	78	1.79 ± 0.77	11.02 ± 1.25	34.03 ± 1.10	21.58 ± 1.47
Pre-eclampsia	46	2.07 ± 0.96	10.75 ± 1.12	34.20 ± 1.03	21.63 ± 1.45
Severe pre-eclampsia	37	1.84 ± 0.79	11.10 ± 1.15	34.39 ± 1.14	22.01 ± 1.34
*P*	—	>0.05	>0.05	>0.05	>0.05

**Table 3:** Serum 25(OH)D levels in each group.

Grouping	Early pregnancy serum 25(OH)*D* value (ng/ml)	Serum 25(OH)D value in the third trimester of pregnancy (ng/ml)	△25(OH)D value (ng/ml)
Normal pregnancy group (D group)	18.21 ± 6.73	21.04 ± 7.63	2.83 ± 4.23
Hypertension during pregnancy (A group)	17.47 ± 6.41	20.66 ± 7.06	3.20 ± 4.65
Preeclampsia group (B group)	14.33 ± 5.60	16.54 ± 6.51	2.20 ± 5.02
Severe pre-eclampsia group (C group)	11.26 ± 4.54	13.03 ± 5.79	1.77 ± 5.07
*F*	15.34	16.26	
*P*	<0.05	<0.05	P'<0.05

## Data Availability

No data were used to support this study.
